This article has been retracted.

# Toxicological Effects of Sewage Water on Chick Embryonic Development

**DOI:** 10.1155/2022/6859798

**Published:** 2022-05-12

**Authors:** Sana Khan, Hafiz Muhammad Noman Baqa, Hamas Mahmood, Muhammad Farooq, Khizar Samiullah, Riffat Yasin, Muhammad Amjad Bashir, Abdur Rahman, Tahir Mehmood, Sagheer Atta, Afrah Fahad Alkhuriji

**Affiliations:** ^1^Department of Zoology Faculty of Sciences Ghazi University Dera Ghazi Khan Punjab, Pakistan; ^2^Hospital Bahawalnagar Punjab, Pakistan; ^3^Hospital Kallurkot Bhakkar Punjab, Pakistan; ^4^Faculty of Veterinary and Animal Sciences, MNSUA, Multan, Pakistan; ^5^Department of Plant Protection Faculty of Agricultural Sciences Ghazi University Dera Ghazi Khan Punjab, Pakistan; ^6^Department of Animal Sciences, University of Veterinary and Animal Sciences, Jhang, Pakistan; ^7^Department of Animal Nutrition, Afyon Kocatepe University, Turkey; ^8^Centre for Applied Molecular Biology (CAMB), University of the Punjab, Lahore-53700, Punjab, Pakistan; ^9^United States Department of Agriculture, Washington DC, USA; ^10^Zoology Department College of Sciences, King Saud University, Riyadh, Saudi Arabia

## Abstract

For toxicity research, a total of 100 fertilized nonincubated eggs were used for this study. There were two trials in this experiment which were further divided into 2 phases based on a different days of sewage water treatment and observation days. In each trial, 50 eggs were used and divided into 5 groups. Group A, B, and C were treated with three different concentrations of pure and diluted sewage water (100%, 70%, and 30%), respectively. Control group D was given 0.3 ml saline solution (0.9% NaCl) and group E was uninjected. Different parameters such as the embryo's body weight, body length, forelimb length, hindlimb length, and head diameter were determined. In trial 1, eggs were treated with sewage water on 7^th^ day of incubation and opened on 8^th^ day (phase I) and 9^th^ day (phase II). When the trial 1 (phase I) findings were compared to the control groups, it was observed that body weight, body length, forelimb length, and hindlimb length were highly statistically significant differences (*p* < 0.01), but the head diameter was not significant (*p* > 0.05). Phase II result showed embryo's head diameter was a highly statistically significant difference (*p* < 0.01), whereas forelimb length was significant (*p* < 0.05), and body weight, body length, and hindlimb length were nonsignificant (*p* > 0.05). In trial 2, eggs were treated with sewage water on 14^th^ day of incubation and opened on 15^th^ day (phase I) and 16^th^ day (phase II). Results of 15^th^ day showed a highly statistically significant (*p* < 0.01) difference in hindlimb length, while body weight, body length, forelimb length, and head diameter were nonsignificant (*p* > 0.05). Phase II of trial 2 showed that on 16^th^ day, body weight, body length, forelimb length, hindlimb length, and head diameter showed a nonsignificant (*p* > 0.05) difference between experimental and control groups. Embryos were observed to be deforming on the 9^th^ day (after 48 hours of exposure to sewage water). Other phases showed no signs of deformation. Except on 8^th^ day of incubation, dose-related mortalities were present in experimental groups, while the control group showed no mortality.

## 1. Introduction

Sewage water, also known as domestic wastewater, is a form of waste water. It is made up of a community of individuals. It is identified by its appearance, organic and inorganic compounds, toxic elements, and the nature of pathogens like bacteria and viruses for example hepatitis A, enteroviruses, protozoa, and parasitic helminths (WHO and UNICEF, [1]). A large proportion of it is made up of greywater (from showers, bathtubs, pools, dishwashers, and cloth washers), black water comes from toilets, along with the human waste washed away, soaps and detergents, and toilet papers (Jackson and Ord, [2]). Untreated sewage water is generated in large quantities across the world, leading to widespread water pollution, particularly in low-income countries. According to UNDP and UN-Habitat figures, 90 percent of all waste water is released untreated into the environment (Corcoran et al., [3]).

With population growth, urbanization, and better living standards, the amount of wastewater produced by domestic, industrial, and commercial sources has increased (Qadir et al., [4]). Sewage water also contains pharmaceutical contaminants that are persistent in the environment. Sewage has also been examined to ascertain the relative rates of prescription and illicit drug use among city residents (Castiglioni et al., [5]). It is also possible to infer general socioeconomic demographics (Choi et al., [6]). However, sewage water can contain biological hazards such as bacteria, viruses, and protozoa, as well as chemical hazards, primarily heavy metals (Hussain et al., [7]). Nowadays, a large amount of untreated sewage/industrial water is being discharged into surface bodies for disposal. It has been indicated that long-term exposure to Cd (heavy metal) in food and water leads to abnormalities in embryonic development (Lone et al., [8]).

Because of a scarcity of water and chemical fertilizer application in many developing countries, using sewage water to irrigate agricultural land is common practice with a long background (Zhang et al., [9]). Many domestic and wild animal species, including other forms of human waste, can use greywater supplies if they are available, raising the risk of pathogen fallout and chemical contamination. This is especially significant in dryland areas where greywater can attract water-dependent animals in an area where groundwater is scarce. Animals consuming greywater infected with animal microbes can promote the transmission of antibiotic-resistant microbes from humans to animals, directly leading to the resistant bacteria in the setting (Alexander and Godrej, [10]). The absence of effective sanitation for human beings is a huge issue. An estimated 4.5 billion cannot get access to appropriate sanitation or do not have access to it at all (WHO and UNICEF, [1]).

Chickens are the most common domestic animal and the primary source of animal protein among domesticated animals (Wang et al., [11]). The chicken model organism has also shown great promise in terms of studying environmental contaminants and chemotherapeutics (Rodriguez et al., [12]). Avian eggs are often used as a bioindicator in environmental pollutant testing systems, and infected eggs can be used to determine the risk of lipophilic environmental pollutants. For more than twenty years, the chicken embryo has been used as a model system for embryology and developmental biology (Stern et al., [13]).

In the present study, the effects of sewage water on the embryonic development of chicks were evaluated. Different parameters such as body weight, body length, forelimb length, hindlimb length, and head diameter were measured. Embryos were also evaluated for normal development. And the mortality rate of developing embryos was also observed.

## 2. Material and Methods

The experiment was performed at Ghazi University's Zoology departmental lab in DG Khan, Punjab, Pakistan. The study was fundamental and experimental. Toxicological effects of sewage water were evaluated in chick embryos in this study. The eggs were purchased from Govt. Poultry Farm Bahawalpur, Punjab, Pakistan. Different concentrations of sewage water were given to experimental groups and compared to control groups. The shells of all the eggs were sterilized with 70% ethanol. With an egg driller, a tiny hole was created in the shell of each egg excepting uninjected eggs. With the small injector, a single dose of each concentration was injected into the air sac of each egg. The hole was sealed with paraffin wax after sewage water had been administered. To ensure the continuity of the embryos, eggs were put in the incubator with the sharp ends pointing down. Eggs were accessible at the times needed. The incubator was maintained at a steady temperature of 37.8°C ± 0.2°C with a humidity of 60-70%. During the incubation cycle, the eggs were automatically rolled at a 45-degree angle to the vertical axis every 2 hours.

### 2.1. Sewage Water Sample Locality

The noncentralized treated sewage water was obtained from Bhutta Colony Dera Ghazi Khan. Dera Ghazi Khan is a district in Pakistan's Punjab province. This sample was collected from house holding tanks.

### 2.2. Sewage Water Sample Analysis

The physical, chemical, and bacteriological properties of sewage water samples were examined at the Laboratory of Pakistan Council of Research in Water Resources (PCRWR) Water Quality Laboratory, Dera Ghazi Khan Punjab, Pakistan.

#### 2.2.1. Physical and Chemical Analyses

Total dissolved solids, electrical conductivity, turbidity, and pH of the water were examined as significant physical parameters in the physical analysis. In chemical analysis, essential chemical parameters such as carbonates, bicarbonates, chloride, calcium, sodium, and potassium were examined. These physicochemical parameters were examined by different methods and instruments as described in Table 1. With the help of this analysis, the following results were obtained from the sewage water sample as shown in Table 2. According to the results of these physical and chemical parameters, it was concluded that sewage water contains various concentrations of contaminants that cause adverse effects on human health and the environment.

#### 2.2.2. Bacteriological Analysis

Total coliform, fecal coliform, and E. coli were studied in the raw form (100%) of sewage water in this sort of examination.  Table 3 displays their results

### 2.3. Experimental Design

A total of 100 fertilized nonincubated eggs (*Gallus gallus domesticus*) were used for this study. There were two trials in this experiment based on different days of sewage water administration. In each trial, 50 eggs were used and divided into 5 groups A, B, C, D, and E. In experimental groups, *A* = 100% sewage water, *B* = 70% sewage water, and *C* = 30% sewage water (0.3 ml dose) were given. Control group D was treated with 0.3 ml saline solution (0.9% NaCl) and E remained uninjected. Each trial was further divided into 2 phases based on different observation days.

- Trial no. 1

For this trial, 50 fertilized eggs were used. These eggs were divided into five groups, each with five eggs. The trial was divided into 2 phases:

- Phase I: this phase included a total of 25 fertilized eggs. On the 7^th^ day of incubation, sewage water was inserted. On the eighth day of incubation, these eggs were determined to be sacrificed (after 24 hours of injection)
- Phase II: a total of 25 fertilized eggs were used for this phase. Sewage water was injected on 7^th^ day of incubation. These eggs were determined to sacrifice on the 9^th^-day of incubation (after 48 hours of injection)

(ii) Trial no. 2

50 fertilized eggs were used for the second trial. These eggs were divided into 5 groups. Trial 2 was separated into two phases:

- Phase I: this phase requires a total of 25 fertilized eggs. Sewage water was given on 14^th^ day of incubation. These eggs opened on 15^th^ day of incubation (after 24 hours of injection)
- Phase II: a total of 25 fertilized eggs were required for this phase. Sewage water was injected on 14^th^ day of incubation. These eggs were determined to sacrifice on the 16^th^-day of incubation (after 48 hours of injection)

### 2.4. Parameters Studied in Trials 1 and 2

On observing days, the eggs were opened, and the outer shells were scratched up to expose the embryo. The embryos were removed from the albumin using a spoon and put on a petri dish and evaluated their different parameters.

Different parameters were studied:

(i) Body length (mm), forelimb length (mm), hindlimb length (mm), and head diameter (mm) were measured on observation days by using a scale. The embryos' body weight (g) was determined by using a digital electronic balance (model no. FA2204)
(ii) Embryos were observed to find the effect of sewage water on the embryonic development of chicks
(iii) The mortality rate was evaluated on different observation days. Mortality percentage (%) was calculated by using the following formula:
  (1) $$\begin{array}{c} \text{Mortality percentage }\left(\%\right)\text{: }\frac{\text{Dead embryos}}{\text{Total number of embryos}}\times 100 \end{array}$$

### 2.5. Statistical Analysis

Using SPSS version 20.0, the data were statistically analyzed. All of the data was given as group mean ± SE, and one-way ANOVA was used to compare the results to the control. For post hoc analysis, Duncan's multiple range test was used. When the difference between the control and experimental groups was less than 0.05, it was considered significant. If *p* < 0.01, it was considered highly significant.

## 3. Results

### 3.1. Trial No. 1

Trial 1 was divided into 2 phases based on different observation days. Sewage water was given on 7^th^ day of incubation. And eggs were opened after 24 hours of sewage water insertion in phase I and after 48 hours in phase II.

In phase I, the finding of body weight, body length, forelimb length, and hindlimb length according to the effects of sewage water demonstrated a highly statistically significant difference (*p* < 0.05), but head diameter showed nonsignificance (*p* > 0.05) between the experimental and control groups. All these parameters were raised in group E which was the control group, while reduced in experimental groups.  Table 4 depicts the sewage water effect on these parameters.

Phase II findings showed that the impact of various concentrations of sewage water on 9^th^ day embryo's head diameter was a highly statistically significant difference (*p* < 0.01), while forelimb length was significant (*p* < 0.05). Body weight, body length, and hindlimb length showed nonsignificance (*p* > 0.05) between the experimental and control groups as represented in Table 4.

### 3.2. Trial No. 2

Trial 2 was divided into 2 phases based on different observation days. On the 14^th^ day of incubation, sewage water was administered. And eggs were opened after 24 hours of sewage water insertion in phase I and after 48 hours in phase II.

In phase I, Table 5 displays the mean ± SE values of various sewage water treatments in comparison to control groups. Hindlimb length revealed a highly statistically significant (*p* < 0.01) difference between the experimental and control groups, while body weight, body length, forelimb length, and head diameter showed nonsignificance (*p* > 0.05).

On 16^th^ day after 48 hours of sewage water administration (phase II), body weight, body length, forelimb length, hindlimb length, and head diameter showed a nonsignificant difference (*p* > 0.05) between the experimental and control groups. These parameters were increased in the control groups, and head diameter increased in group A, while these values decreased in the experimental groups as depicted in Table 5.

### 3.3. Effect of Sewage Water on Chick Embryos on Different Observation Days

Figure 1 displays the development of various body parts after being exposed to sewage water treatments and compared to control groups. Embryos exhibited normal development in phase I of trial 1; however, deformation of body parts of chick embryos in experimental groups (A, B and C) was detected on the 9^th^ day after 48 hours of sewage water treatment in phase II, as compared to control groups that showed normally developed body parts.

In trial 2, sewage water was given on 14^th^ day of incubation; after 24 hours (phase I) and 48 hours (phase II) of administration, embryos were evaluated for normal development. In both phases, embryos showed no abnormality.

### 3.4. Mortality Percentage (%) on Different Observation Days

Mortality percentage (%) in different experimental and control groups has been given in Figure 2. There was no mortality in 8^th^ day old chick embryos treated with sewage water on 7^th^ day. While in others, mortalities were increased with increasing concentration of sewage water. Control groups did not show any mortality.

## 4. Discussion

The main purpose of this study was to determine the toxicological effects of sewage water on the embryonic development of chicks. A total of 100 fertilized nonincubated eggs (*G. gallus domesticus*) were used for this study. There were two trials in this experiment. Each trial was further divided into 2 phases. In each trial, 50 eggs were used and divided into 5 groups. Groups A, B, and C were treated with three different concentrations of sewage water (100%, 70%, and 30%) and compared to controls (saline solution given 0.9% NaCl and uninjected group). Different parameters such as body weight, body length, hindlimb length, forelimb length, and head diameter were evaluated on the 8^th^, 9^th^, 15^th^, and 16^th^ days.

When examined, sewage water included total coli, fecal coli, and E. coli. Hughes and Thompson (2004) had also found that total coliforms (which include *Enterobacteriaceae* and fecal coliforms) are the most common bacteria and are used as indications of sewage pollution.

Greywater (from showers, bathtubs, pools, dishwashers, and clothes washers) makes up a major amount of sewage water, as does black water (from toilets, along with the human waste washed away, soaps and detergents and toilet papers). Greywater, according to Jackson and Ord, is water that is of poor significance than potable water (drinking water) but of greater value than black water (Jackson and Ord, [2]). In the current investigation, the sewage water analyzed was grey and had a foul smell.

When sewage water was examined in the current study, it included nitrate 0.95 mg/l and sodium 680 mg/l, which affected the body weight of chick embryos in trials 1 and 2, except in phase II of trial 1, in which its value decreased in control group E. This work was supported by the work of (Mohamadi et al., [14]) who found that adding nitrate sodium to the air sac of fertilized chicken eggs did not affect the production, hatching, or survival of one-day chicks. However, it promotes hypoxia, diminishes overall antioxidant capacity, and increases malondialdehyde in the body, resulting in a reduction in freshly chick weight. Grizzle et al. [15] had found that water quality in broiler farms has a negative impact on broiler performance, which is negatively associated with body weight and immune resistance.

In the present study, body length decreased in chick embryos in the sewage water-treated groups when compared with the control groups. The present study was in corroboration with the findings of (Bhanot and Hundal, [16]) that conducted an experiment on fish *Labeo rohita* and found a decrease in total body length in the sewage water-treated groups in comparison with the control. The present study was also consistent with (Sultana et al., [17])'s findings who had also observed a decrease in the morphometric parameters, such as total body length and standard length of the fish *Labeo rohita* which was inhabiting industrial wastewater contaminated water of river Ravi, Pakistan.

Mortalities had occurred in all experimental groups except on the 8^th^ day of incubation (phase I of trial 1). After 24 hours of sewage water treatment, there was less mortality that occurred in chick embryos. The dose-dependent mortality rate was present in the current investigation, and the mortality rate grew progressively as the sewage water concentration was raised (100% sewage water). It was in line with the findings of (Miniawy et al., [18]) who found dose-dependent mortality rate in broiler chicks was present.

The present study showed no mortality in control groups in all trials. It was not supported by the findings of (Kalita et al., [19]) who reported that different aspects, including air shortage, egg size, genetic makeup, breeding, pathological circumstances, lack of basic cleanliness, and the arrangement of the eggs throughout incubation, as well as the alignment of the primitive streak, may be involved in the mortality of embryos in control groups.

## 5. Conclusion

Sewage water not only affects the chickens but also had a detrimental effect on chick embryos. Sewage water penetrates the egg and may affect the chick embryo's development when given at an early stage or later stage of development. It may cause a decrease in body weight, and body length, along with the forelimb and hindlimb length of chick embryos. Sewage water also caused mortality in chick embryos. The mortality rate was increased in a dose-dependent manner, particularly after 48 hours of exposure to sewage water. Pollutants in sewage water cause low chicken output. It was concluded that chickens should be provided with clean water and raised in sanitary conditions.

## Figures and Tables

**Figure 1:** Effect of sewage water in different sewage water-treated groups (groups A–C) and control groups (groups D and E): (a) chick embryos on 8^th^ day given sewage water on 7^th^ day of incubation, (b) chick embryos on 9^th^ day administered sewage water on 7^th^ incubation day, (c) chick embryos on 15^th^ incubation day given sewage water on 14^th^ day of incubation, and (d) Chick embryos on 16^th^ day injected sewage water on 14^th^ day of incubation.

**Figure 2:** Mortality percentage (%) in different sewage water-treated groups and control groups on different observation days.

**Table 1:** Methods/instruments for physical and chemical parameter analysis.

Sr. no.	Parameters	Analysis methods/instruments
1.	pH	pH meter
2.	Electrical conductivity	Conductivity method, electrical conductivity meter
3.	Turbidity	Turbidity meter/nephelometer
4.	Color	Sensory test
5.	Carbonates	Titration (standard solution of strong acid)
6.	Bicarbonates	Titration (standard solution of strong acid)
7.	Alkalinity	Titration (standard solution of strong acid)
8.	Calcium	Calcium meters
9.	Chloride	Titration (silver nitrate solution)
10.	Fluoride	Fluoride electrode method (water+zirconyl xylenol orange complex reagent)
11.	Hardness	Titration (standard solution of strong acid)
12.	Magnesium	EDTA (ethylenediaminetetraacetic acid)
13.	Sodium	Flame photometer
14.	Nitrate	Visible spectrophotometer
15.	Potassium	Flame photometer
16.	Sulfate	Titration (barium chloride)
17.	TDS	TDS meter

**Table 2:** Results of physicochemical parameter analysis.

Sr. no.	Physicochemical parameters	Results
1.	Appearance	Turbid
2.	Color	Greyish
3.	Odor	Foul
4.	Bicarbonate (mg/l)	165
5.	Alkalinity (mmol/l)	3.3
6.	Calcium (mg/l)	426
7.	Carbonate	Nil
8.	Chloride (mg/l)	208
9.	Conductivity	7560
10.	Turbidity	225
11.	Fluoride (mg/l)	3.65
12.	Hardness (mg/l)	1425
13.	Magnesium (mg/l)	87.48
14.	Nitrate	0.95
15.	pH	8.25
16.	Potassium (mg/l)	22
17.	Sodium (mg/l)	680
18.	Sulfate (mg/l)	3685
19.	TDS (mg/l)	4536

**Table 3:** Results of bacteriological analysis.

Sr. no.	Parameters	Results
1.	Total coli form	210
2.	Fecal coli form	112
3.	E. Coli	75

**Table 4:** Different parameter's mean ± standard error of chick embryos given sewage water on 7^th^ day of incubation.

Parameters	Trial 1	Observation days	Experimental groups			Control groups		*p* value
			A	B	C	D	E	
Body weight (g)	Phase I	8^th^ day	0.37 ± 0.07^b^	0.69 ± 0.34^b^	0.42 ± 0.05^b^	1.43 ± 0.16^a^	1.74 ± 0.03^a^	0.01^∗∗^
	Phase II	9^th^ day	1.42 ± 0.06	1.22 ± 0.08	1.47 ± 0.03	1.28 ± 0.11	1.16 ± 0.09	0.14
Body length (mm)	Phase I	8^th^ day	24.00 ± 1.58^b^	21.60 ± 1.16^b^	22.00 ± 1.14^b^	33.00 ± 2.19^a^	33.40 ± 1.07^a^	0.01^∗∗^
	Phase II	9^th^ day	31.00 ± 1.52	30.75 ± 1.10	32.50 ± 1.04	31.40 ± 1.07	31.20 ± 0.58	0.80
Forelimb length (mm)	Phase I	8^th^ day	5.60 ± 0.87^ab^	3.60 ± 0.81^b^	4.00 ± 0.70^b^	6.40 ± 0.748^a^	7.20 ± 0.37^a^	0.01^∗∗^
	Phase 2	9^th^ day	6.33 ± 0.33^b^	7.75 ± 0.47^ab^	7.62 ± 0.68^ab^	9.40 ± 0.92^a^	9.40 ± 0.24^a^	0.02∗
Hindlimb length (mm)	Phase I	8^th^ day	9.00 ± 0.83^b^	5.80 ± 0.73^c^	8.00 ± 1.04^bc^	10.00 ± 1.0^ab^	12.00 ± 0.70^a^	0.01^∗∗^
	Phase II	9^th^ day	12.00 ± 1.52	11.00 ± 0.70	13.25 ± 1.54	14.00 ± 1.73	13.60 ± 0.60	0.49
Head diameter (mm)	Phase I	8^th^ day	4.60 ± 0.24	3.40 ± 0.67	3.40 ± 0.50	4.60 ± 0.67	5.40 ± 0.40	0.06
	Phase II	9^th^ day	3.66 ± 0.33^b^	7.00 ± 0.40^a^	7.00 ± 0.70^a^	6.60 ± 0.40^a^	7.00 ± 0.31^a^	0.01^∗∗^

^a, b, c^Values with a different superscript in row differ significantly (^∗^*p* < 0.05, ^∗∗^*p* < 0.01).

**Table 5:** Different parameter's mean ± standard error of chick embryos given sewage water on 14^th^ day of incubation.

Parameters	Trial 2	Observation days	Experimental groups			Control groups		*p* value
			A	B	C	D	E	
Body weight (g)	Phase I	15^th^ day	8.67 ± 1.14	9.56 ± 0.99	11.05 ± 0.37	11.27 ± 0.36	10.87 ± 0.18	0.10
	Phase II	16^th^ day	15.58 ± 1.23	15.07 ± 2.14	14.80 ± 0.63	21.93 ± 5.32	18.28 ± 2.26	0.32
Body length (mm)	Phase I	15^th^ day	6.15 ± 0.33	6.26 ± 0.32	6.75 ± 0.10	6.35 ± 0.26	6.38 ± 0.11	0.56
	Phase II	16^th^ day	7.66 ± 0.35	6.85 ± 0.59	6.77 ± 0.15	7.73 ± 0.37	7.60 ± 0.32	0.29
Forelimb length (mm)	Phase I	15^th^ day	2.10 ± 0.24	2.54 ± 0.17	2.17 ± 0.21	1.92 ± 0.09	2.44 ± 0.12	0.12
	Phase II	16^th^ day	2.96 ± 0.03	2.60 ± 0.23	2.80 ± 0.12	3.10 ± 0.20	2.96 ± 0.24	0.42
Hindlimb length (mm)	Phase I	15^th^ day	2.62 ± 0.11^b^	2.98 ± 0.03^a^	3.20 ± 0.07^a^	3.17 ± 0.16^a^	3.14 ± 0.07^a^	0.01^∗∗^
	Phase II	16^th^ day	4.00 ± 0.05	3.45 ± 0.55	4.07 ± 0.11	4.43 ± 0.34	4.56 ± 0.12	0.20
Head diameter (mm)	Phase I	15^th^ day	2.10 ± 0.62	2.54 ± 0.50	2.17 ± 0.75	1.92 ± 0.47	2.44 ± 0.37	0.13
	Phase II	16^th^ day	8.66 ± 0.88	8.25 ± 1.03	8.00 ± 0.91	8.50 ± 1.89	8.16 ± 0.83	0.99

^a, b, c^Values with different superscripts in row differ significantly (^∗^*p* < 0.05, ^∗∗^*p* < 0.01).

## Data Availability

All data are available within manuscript, and additional data will be provided on request.
